RETRACTED

# Lipoma Growing on the Back for 26 Years: A Bizarre Case Report

**DOI:** 10.7759/cureus.56999

**Published:** 2024-03-26

**Authors:** Samiksha V Gupta, Shubham Durge, Nachiket P Rahate, Prashant V Rahate

**Affiliations:** 1 Psychiatry and Behavioral Sciences, Jawaharlal Nehru Medical College, Datta Meghe Institute of Higher Education and Research, Wardha, IND; 2 General Surgery, Jawaharlal Nehru Medical College, Datta Meghe Institute of Higher Education and Research, Wardha, IND; 3 Surgery, Seven Star Hospital, Nagpur, IND

**Keywords:** suction-assisted lipectomy, histopathology, surgical skin excision, benign, lipoma

## Abstract

Lipoma is one of the most typical and benign tumors. They are typically regarded as a mass that is painless, asymptomatic, and slow-growing. It is composed of fat cells of the adult type. It can occur anywhere in the body and is often called a "universal" or ubiquitous tumor. They can develop in any region containing adipose tissue, with a higher prevalence in the subcutaneous tissue of the trunk and the nape of the neck and the limbs and occasionally in other locations, including the hand. There are three main varieties: encapsulated, diffuse, and multiple lipomas. A few lipomas may contain other tissues: fibrolipoma, neurolemma, and myelolipoma. Lipoma, when present for a long time, may undergo certain changes. This is particularly true in cases of lipoma under subcutaneous tissues of the thigh, buttock, or retroperitoneal lipoma. Such changes can be malignant, sarcomatous, calcification, or saponification. Clinically, a lipoma can occur in different anatomical situations; according to this, a lipoma can be classified into subcutaneous type, subfascial type, intramuscular type, subserous type, submucous type, intra-articular type, or it can be intraglandular. Lipomas, the most prevalent benign mesenchymal tumors, consist of mature lipocytes. Typically, lipomas are small, weighing only a few grams, with a maximum diameter usually under 2 cm. The term "giant" is applied when a lipoma reaches a diameter of at least 10 cm or weighs a minimum of 1,000 g. Due to their substantial size, giant lipomas can lead to functional limitations, such as lymphedema, pain syndromes, or nerve compression. Given the unique nature of this condition, characterized by the considerable size of the lesion and the challenges in both diagnosis and treatment, we present a case involving a 45-year-old woman with a giant lipoma in the suprascapular region.

## Introduction

Lipomas are prevalent noncancerous tumors in soft tissues, typically small and benign. Nonetheless, large lipomas are infrequent, and their size may lead to discomfort and nerve compression syndrome. A lipoma is a slow-growing, fatty lump generally situated between the skin and the underlying muscle layer. Lipomas, with a doughy texture and usually nontender, exhibit easy mobility under slight finger pressure. These growths are commonly discovered during middle age, and some individuals may experience the development of multiple lipomas. Importantly, lipomas are benign and pose no cancer risk [1].

RETRACTED

Lipomas are noncancerous growths composed of fat cells (adipocytes), appearing as soft, painless masses predominantly found on the trunk but potentially occurring anywhere on the body. Typically, lipomas vary in size, ranging from 1 cm to greater than 10 cm. These growths are categorized as mesenchymal tumors and can manifest in areas of the body where regular fat cells are present. In a minority of cases, approximately 2% to 3% of affected individuals, there may be a genetic component, with multiple lesions inherited in a familial pattern [2]. 

In certain solitary lipomas, a gene association has been identified on chromosome 12, where some tumors exhibit a mutation in the HMGA2-LPP fusion gene [3]. Additionally, various genetic syndromes manifest lipomas as a clinical feature. A 45-year-old female patient complaining of a massive swelling over the right upper back of the supraclavicular region was diagnosed with lipoma. Ultrasonography (USG) of the swelling showed a homogenous soft-tissue mass in the suprascapular region, suggestive of lipoma. Histologically, the lesion comprised multilobulated, mature adipose cells, leading to a benign lipoma diagnosis. The preferred approach for dealing with giant lipomas involves surgical excision to minimize complications, prevent a recurrence, and mitigate potential harm from the benign giant tumor compressing major vessels or nerves. This strategy aims to enhance local control and ensure an accurate final diagnosis.

## Case presentation

A 45-year-old female patient came to a tertiary care clinic in the city of Wardha with complaints of massive swelling over the right side of her upper back in the suprascapular region. The patient reported difficulty in wearing clothes and felt embarrassed about the swelling cosmetically. The patient noticed the swelling 26 years back but did not heed it. The patient has no significant family history of such swelling. Upon examination, the patient was afebrile to the touch (37°C) and had a blood pressure of 130/90 mmHg. On local examination, the swelling was approximately 16 x 20 cm in dimensions, freely mobile and firm in consistency; the local temperature was not raised; and the skin color over the swelling appeared normal. The patient is not able to recall if any trauma was associated with it. The swelling was not associated with tenderness, ulcer, or sinus discharge. On local examination, the slip sign was positive, suggesting a diagnosis of lipoma, as seen in Figure 1

**Figure 1:** The image depicts a giant lipoma over the right suprascapular region.

RETRACTED

Upon further investigation, her blood glucose level was 110 mg/dl, and further investigation is listed in Table 1.

**Table 1:** All the values are within the normal range, suggesting no infection or inflammation. RBC: Red blood cell; WBC: white blood cell The values are according to source [4].

Test	Observed values	Reference values
Hemoglobin	11.5 mg/dl	10-15 mg/dl
RBC counts	4.45 mcL	3.92-5.15 mcL
Platelet counts	100,000/mm^3^	150,000-450,000/mm^3^
WBC counts	7,500 cells/mm^3^	4,000-11,000 cells/mm^3^
Eosinophils	1%	0%-6%
Basophils	0%	0%-2%
Neutrophils	58%	50%-62%
Monocytes	9%	0%-10%
Lymphocytes	32%	20%-40%

On USG of the local site, the lesion shows a well-defined swelling, encapsulated, 16 x 20 cm in the subcutaneous plane on the right suprascapular region, with no calcification and minimal to no vascularity on Doppler. The fine-needle aspiration cytology (FNAC) of the mass revealed adipocytes displaying large, univacuolated dark cytoplasm and eccentric nuclei, aligning with the clinical diagnosis of lipoma. No cellular atypia or malignancy was observed. Consequently, a complete surgical excision was performed, and intraoperatively, no neuromuscular involvement was detected, as seen in Figure 2.

**Figure 2:** The image shows a complete excision of the giant lipoma.

The preoperative procedure of lipoma excision was explained to the patient and her relatives, and consent was acquired for the same. The patient was kept nil per oral overnight. The tumor was completely surgically excised using an arcuate incision. Subsequently, the detachment was carried out anteriorly and posteriorly using fingers, followed by enucleation after ligation of the nourishing pedicle, as seen in Figure 3.

**Figure 3:** Intraoperative image of enucleation of lipoma.

Excess skin was resected to facilitate aesthetic closure, and a suction Redon drain was employed. The procedure proceeded without any complications, and the patient was subsequently transferred back to the ward. Dressing changes were performed regularly. The excised piece measured 16 cm by 20 cm and weighed 2200 g. The postoperative course was uneventful, and the drain was removed on the second day after the surgery. The histological examination of the surgical specimen confirmed the diagnosis of a fibrolipoma, ruling out any signs of malignancy as seen in Figure 4. During the six-month follow-up, there were no indications of recurrence in the patient.

RETRACTED

**Figure 4:** Histopathological slide, visualized under 40x magnification and stained by hematoxylin and eosin stain, showing mature adipocytes with fibrous strands suggestive of fibrolipoma.

## Discussion

Superficial subcutaneous lipoma is highly prevalent, constituting 15% to 40% of all soft tissue tumors. Typically affecting individuals in middle age, there is no gender predilection when the lipoma is solitary. These growths can manifest anywhere on the body, with approximately 10% to 15% occurring on the back [5]. The etiopathogenesis of lipomas remains poorly understood, potentially attributed to minimal and repetitive trauma. In 5% to 15% of instances, lipomas occur in multiple forms, showing a male predominance. About a third of these cases involve hereditary transmission, often following an autosomal dominant pattern called multiple familial lipomas. Typically emerging between the ages of 30 and 50, these lipomas manifest in the subcutaneous tissue of the limbs and trunk, with a tendency to spare the neck and shoulders. Some theories suggest a link with obesity, although conclusive evidence is lacking [6].

When completely excised, extending to healthy surrounding areas, these lipomas typically do not undergo degeneration. However, achieving complete excision can be challenging, especially in the case of deep-seated lipomas. Lipomas often present as asymptomatic, as observed in our patient. However, some individuals may experience vague pain, tension, or compression of a peripheral nerve associated with the presence of lipomas. The primary concern is typically aesthetic, given lipomas' massive and unsightly nature. However, functional discomfort, as seen in our patient, should not be underestimated, as lipomas can lead to issues such as skin macerations, nerve compression, and an abnormal spinal posture. Clinical examination is key in guiding the diagnosis, with lipomas commonly presenting as painless, soft, regular, and mobile tumors. In our specific case, due to the tumor's size exceeding 10 cm, FNAC was recommended. This procedure was performed to confirm the benign nature of the tumor. FNAC is recognized as a cost-effective and rapid method for diagnosing lipomas with high accuracy, boasting a sensitivity of 94% and specificity of 97% [7]. The standard imaging modality for lipomas is USG. Magnetic resonance imaging (MRI) may rule out malignancy such as liposarcoma. Given the rare occurrence of liposarcoma (2.4 per million per year), an MRI is advisable only in cases with strong clinical indications, including significant size, rapid growth, pain, ulceration, increased vascularity, and immobility.

RETRACTED

Liposuction and suction-assisted lipectomy have recently emerged as potential alternative treatments for giant lipomas, offering cosmetic benefits. However, this approach has potential drawbacks, including challenges in visualizing the tumor, specimen fragmentation complicating histopathological analysis, and an increased risk of recurrence due to incomplete resection [8]. Differential diagnosis considerations include other soft tissue tumors like ganglion cysts, giant cell tumors, myxomas, angiolipomas, intraneural lipofibroma, and liposarcoma [9].

## Conclusions

Despite its benign nature, giant lipomas frequently cause notable functional discomfort, and the primary treatment approach is surgical. Surgeons often harbor concerns about potential malignant degeneration. Malignancy should be suspected in cases exhibiting clinical features such as significant size, rapid growth, pain, and immobility. Imaging techniques such as USG, MRI, and cytopathology should be employed to confirm the diagnosis and exclude malignancy. In situations where histology may not always be readily available, opting for primary excision surgery in cases with a strong suspicion of lipoma, coupled with a systematic anatomopathological study of the surgical specimen, is advised.
